This article has been retracted.

# Effect of miR-195-5p on cardiomyocyte apoptosis in rats with heart failure by regulating TGF-β1/Smad3 signaling pathway

**DOI:** 10.1042/BSR20200566

**Published:** 2020-05-12

**Authors:** Chun Xie, Huaxin Qi, Lei Huan, Yan Yang

**Affiliations:** 1 Department of Cardiology, Jinan People's Hospital Affiliated to Shandong First Medical University, Jinan City 271199, Shandong Province, China; 2 Health Examination Center, Qilu Hospital of Shandong University, Jinan City 250012, Shandong Province, China

**Keywords:** miR-195-5p, TGF-β1/Smad3 signaling pathway, heart failure rats, cardiomyocyte, apoptosis

## Abstract

**Purpose:** The present study set out to investigate the effect of miR-195-5p on cardiomyocyte apoptosis in rats with heart failure (HF) and its mechanism.

**Methods:** HF rat model and hypoxia/reoxygenation (H/R) cardiomyocyte model were established. miR-195-5p expression and transforming growth factor-β1 (TGF-β1)/signal transduction protein (Smad)3 signaling pathway in HF rats and H/R cardiomyocytes were interfered. miR-195-5p expression was tested by Rt-PCR, TGF-β1/Smad3 signaling pathway related proteins were detected by Western Blot, apoptosis of HF rat cardiomyocytes was tested by TUNEL, and apoptosis of cardiomyocytes induced by H/R was checked by flow cytometry.

**Results:** miR-195-5p was lowly expressed in myocardium of HF rats, while TGF-β1 and Smad3 proteins were high-expressed. Up-regulating miR-195-5p expression could obviously inhibit cardiomyocyte apoptosis of HF rats, improve their cardiac function, and inhibit activation of TGF-β1/Smad3 signaling pathway. Up-regulation of miR-195-5p expression or inhibition of TGF-β1/Smad3 signaling pathway could obviously inhibit H/R-induced cardiomyocyte apoptosis. Dual-luciferase reporter enzyme verified the targeted relationship between miR-195-5p and Smad3.

**Conclusion:** miR-195-5p can inhibit cardiomyocyte apoptosis and improve cardiac function in HF rats by regulating TGF-β1/Smad3 signaling pathway, which may be a potential target for HF therapy.

## Introduction

Heart failure (HF) is a complex clinical syndrome in which the ejection or filling ability of left ventricle is damaged due to cardiac structure or dysfunction. HF is usually the final stage of various cardiovascular diseases [1,2]. Recently, with the changes of social environment and living habits, incidence of cardiovascular diseases is also getting higher and higher, and almost any cardiovascular disease will eventually lead to the occurrence of HF. Although considerable progress has been made in medical technology, mortality within 5 years after patients are diagnosed as HF is still as high as 50%, which is a great threat to human life and health [3,4].

Apoptosis refers to a kind of spontaneous programmed cell death. Recent studies have found that cardiomyocyte apoptosis may be a crucial part of HF pathogenesis [5]. Previous studies [6] have shown that cardiomyocyte apoptosis is very obvious in patients with HF. Therefore, it is quite significant to explore the mechanism of cardiomyocyte apoptosis in HF patients and how to prevent it for HF treatment. As a non-coding short-chain RNA, miRNA can play a biological regulatory role by combining with target genes. Recently, miRNA has been found to be effective in all kinds of diseases, including cardiovascular diseases [6]. miR-195-5p has been proved to be down-regulated in coronary artery blood flow disorders in the past [7], which suggests that miR-195-5p may be effective in the development and progression of cardiovascular diseases. However, it is not clear whether miR-195-5p can affect cardiomyocyte apoptosis in HF. Previous studies [8] have reported that transforming growth factor-β1 (TGF-β1)/signal transduction protein (Smads) 3 signaling pathway can affect the formation of myocardial fibrosis by regulating transcription of extracellular matrix synthesis genes, and myocardial fibrosis is also one of the major pathological changes of HF. However, some studies [9] have also found that TGF-β1/Smad3 signaling pathway also participates in cardiomyocytes’ apoptosis process. We found a targeted relationship between miR-195-5p and Smad3 through online website prediction, so we speculated whether miR-195-5p could participate in HF’s development and progression by regulating TGF-β1/Smad3 pathway.

Therefore, we established HF rat model to explore miR-195-5p’s effect on cardiomyocyte apoptosis in HF rats and its related mechanisms to provide more target directions for HF prevention and treatment.

## Materials and methods

### Experimental animals and materials

One hundred SD rats (bought from the Experimental Animal Center of Sun Yat-sen University) with body mass of 210–255 g were selected and fed in an environment with temperature of 23–28°C and relative humidity of 45–70%, with normal diurnal rhythm alternating and free to eat and drink. Operation of the modeling process on rats conforms to the standards of the Laboratory Animal Ethics Committee of our hospital. H9c2 cardiomyocytes were bought from Shanghai Cell Bank, Chinese Academy of Sciences. Fetal bovine serum (FBS) and trypsin were bought from HyClone. TGF-β1, Smad3, Bax, Bcl-2, and activated Cle-Caspase-3 monoclonal antibodies were all bought from Cell Signaling, U.S.A. Rabbit anti-human β-actin monoclonal antibody was bought from Proteintech Group, Inc. BCA protein concentration determination kit was purchased from Shanghai Well Biotech Co., Ltd. TUNEL apoptosis detection kit (Roche Diagnostics, Basel, Switzerland), miRNA NC, internal reference U6 and β-actin primer were all synthesized and designed by Shanghai GenePharma Co., Ltd. Real-time quantitative PCR instrument (Bio-Rad, Berkeley, California, U.S.A.), Annexin V-FITC/PI apoptosis kit (BestBio Biotechnology Co., Ltd., Shanghai, China), flow cytometry CytoFLEX LX (Beckman, Brea, California, U.S.A.), DMEM (Gibco, Rockville, MD, U.S.A.). The present study has been approved by the animal experimental ethics committee of Laiwu People’s Hospital. All experiments took place at Laiwu People’s Hospital.

### Establishment of animal model

HF rat model [10] was prepared by abdominal aortic stenosis method. HF was induced by ligating abdominal aorta to create a cardiac load pot. Rats were randomized into blank control group (BCG), sham operation group (SOG), HF group, HF+miR-195-5p-agomir group and miR-NC group, with 20 rats in each group. Those in the BCG were fed conventionally without any treatment, and the rest were anesthetized with 4% isoflurane (KEW Biotechnology Co., Ltd., Nanjing, C002). First, we filled the induction box with anesthetics and put the rats into it. Then, we gently shook the induction box. If the rats turned over and did not try to recover their lying posture, it meant that they had been completely anesthetized [11]. After they were completely anesthetized (approximately 2–3 min), we closed the box. After that, they were fixed on the operation table in supine position. Their heads/noses were placed in the anesthesia mask and fixed with 2% isoflurane as the maintenance dose. Then, we connected them with electrocardiograph, and respiratory support was provided with a small animal ventilator. Then skin preparation, disinfection, and laparotomy were carried out on the rats in a sterile environment. After laparotomy, the abdominal aorta was explored and blunt separation was carried out on the abdominal aorta above the right kidney. The abdominal aorta was ligated with needle No.7, and then the incision was sutured and closed. Four weeks after modeling, the rats in the HF+miR-195-5p-agomir group were injected with 100 μl of miR-195-5p-agomir (the solvent was physiological saline, 100 nmol/ml) via caudal vein, those in the HF group were injected with 100 μl of miR-NC (the solvent was physiological saline, 100 nmol/ml) via caudal vein, and those in the SOG were injected with the same dose of physiological saline via caudal vein twice a week; their cardiac function were detected 4 weeks after treatment, and they were anesthetized according to the above methods and killed for cervical dislocation for subsequent related detection. The animal experiment was conducted in accordance with the ‘Guidelines for the Management and Use of Experimental Animals’ of the United States, and this experiment has been declared by animal experiment ethics.

### Cardiac function test

Four weeks after treatment, cardiac function of the rats was tested. First, hair on their left anterior chest was cleaned. Then, the cardiac function was measured vis echocardiography (Vevo2100, VisualSonics), and the left parasternal long-axis was detected. The detection indexes included interventricular septal end-diastolic thickness (IVSd), interventricular septal end-systolic thickness (IVSs), left ventricular end-diastolic inner diameter (LVIDd), left ventricular end-systolic inner diameter (LVIDS), and ejection fraction (EF%).

### Cardiomyocyte apoptosis in myocardium detected by TUNEL

Heart tissue was fixed 24 h with 4% formaldehyde at room temperature, washed with PBS, dehydrated, embedded with paraffin and cut into 4-μm-thick slices, and then apoptotic myocardial cells were detected in strict conformity with the instructions of the detection kit. Cells with brown stained nuclei-manifested apoptotic cells and were counted in five microscope fields under fluorescence microscope. Ratio of TUNEL-positive cells to total myocardial cells was calculated.

### Establishment of cell model

Cardiomyocyte apoptosis was induced by establishing hypoxia/reoxygenation (H/R) model of cardiomyocytes, and miR-195-5p and TGF-β1/Smad3 signaling pathway’s effects on cardiomyocyte apoptosis were observed. H9c2 cells were put in DMEM (containing 10% FBS) and incubated at 37°C, 5% CO_2_. When grown to 80%, they were collected and divided into BCG, H/R, miR-195-5p-mimics group, miR-NC group, Si-Smad3 group, and Si-NC group. Those in the BCG were cultured normally. Those in other groups were replaced by DMEM with serum-free and sugar-free medium, and they were cultured in a hypoxia incubator at 37°C, 94% N_2_ and 5% CO_2_. After 24 h, they were transferred to a medium containing 10% FBS, and incubated 3 h at 37°C, 5% CO_2_ to establish an H/R model. After the model was established, miR-195-5p-mimics, miR-NC, Si-Smad3, and Si-NC were transfected into the cells 24 h via Lipofectamine 2000, while those in the H/R group were not transfected.

### Rt-PCR detection

The total RNA in tissues and cells was extracted with TRIzol reagent, and its purity and concentration were detected by ultraviolet spectrophotometer. Then, 5 μg of total RNA was taken respectively to reverse transcribe cDNA according to the instructions of the kit. The reaction parameters were as below: 37°C for 15 min, 42°C for 35 min, 70°C for 5 min. PCR amplification was carried out after reverse transcription. PCR conditions were as follows: pre-denaturation at 94°C for 45 s, denaturation at 94°C for 10 s, annealing extension at 60°C for 45 s, a total of 40 cycles and three experiments. miR-195-5p employed U6 as the internal reference and the data were analyzed via 2^−△△*c*_q_^ [12].

### Western blot test

Myocardium and cultured myocardial cells were collected to extract total protein by RIPA lysis method. Protein concentration was detected by BCA method and adjusted to 4 μg/μl. It was then under 12% SDS/PAGE electrophoresis separation, and transferred to PVDF membrane after ionization. It was dyed with Ponceau S working solution, soaked 5 min in PBST, washed, and sealed 2 h with 5% defatted milk powder. Bax (1:500), Bcl-2 (1:500), Cle-Caspase-3 (1:500), TGF-β 1 (1:1000), Smad 3 (1:1000), and β-Actin primary antibody (1:500) were supplemented to block them all night long at 4°C. The membrane was washed to remove primary antibody, horseradish peroxidase labeled goat anti-rabbit secondary antibody (1:1000) was supplemented, and it was incubated 1 h at 37°C, rinsed three times with PBS, each time for 5 min. The protein bands on the membrane were developed in a dark room via the enhanced chemiluminescence (ECL) reagent, and the excess liquid was absorbed with a filter paper.

### Cardiomyocyte apoptosis detected by flow cytometry

Transfected cells were digested with 0.25% trypsin, cleaned twice with PBS after digestion, added with 100 μl of binding buffer, prepared into 1 × 10^6^/ml suspension, sequentially added with AnnexinV-FITC and PI, incubated 5 min in dark at room temperature, and detected with FC500MCL flow cytometry. The test was repeated three times and results were averaged.

### Detection of dual-luciferase reporter enzyme

Targetscan7.2 was employed to predict miR-195-5p downstream target genes. Smad3-3′UTR wild-type (Wt), Smad3-3′UTR mutant (Mut), miR-195-5p-mimics and miR-NC were transferred into H9c2 cells by Lipofectamine™ 2000 kit, and luciferase activity was tested by dual-luciferase reporter gene assay kit (Promega) 48 h after transfection.

### Statistical methods

The collected data were statistically analyzed via SPSS20.0 (IBM, Armonk, NY, U.S.A.) software package, and GraphPad 7 software package was adopted to draw the required pictures. Intergroup comparison was under independent-samples *t* test, and multigroup comparison was under one-way analysis of variance, and post hoc pairwise comparison was under LSD *t* test. *P*<0.05 was seen as statistical difference.

## Results

### miR-195-5p expression in myocardium of HF rats and its effect on cardiac function

Compared with rats in the BCG and SOG, miR-195-5p was dramatically down-regulated in the HF group and miR-NC group rats, while its expression in myocardium of rats in the HF+miR-195-5p-agomir group increased markedly (*P*<0.05). Compared with rats in the BCG and SOG, LVIDs, IVSd, IVSs, and LVIDd of those in the HF group were higher, and EF reduced greatly (*P*<0.05). Compared with HF rats, LVIDs, IVSd, IVSs, and LVIDd of those in the HF+miR-195-5p-agomir group reduced obviously, and EF increased obviously (*P*<0.05) (Figure 1).

**Figure 1:** miR-195-5p expression in HF rat myocardium and its effect on cardiac function (**A**) miR-195-5p expression in HF rat myocardium. (**B**–**F**) Effect of miR-195-5p on cardiac function in HF rats. *, ^#^ compared with BCG and SOG (*P*<0.05).

### miR-195-5p overexpression’s effect on cardiomyocyte apoptosis in HF rats

Compared with rats in the BCG and SOG, the cardiomyocyte apoptosis rate of those of the HF group and miR-NC group increased dramatically, the pro-apoptotic protein Bax was remarkably up-regulated and the anti-apoptotic protein Bcl-2 was markedly down-regulated (*P*<0.05). However, compared with HF group rats, the rate of those rats in the HF+miR-195-5p-agomir group reduced dramatically, the Bax was remarkably down-regulated, and Bcl-2 was markedly up-regulated (*P*<0.05) (Figure 2).

**Figure 2:** Effect of miR-195-5p overexpression on cardiomyocyte apoptosis in HF rats (**A**) Effect of miR-195-5p overexpression on cardiomyocyte apoptosis rate in HF rats. (**B**–**D**) Effect of miR-195-5p overexpression on apoptosis-related proteins expression in HF rat cardiomyocytes. *, # compared with BCG and SOG (*P*<0.05).

### miR-195-5p overexpression’s effect on apoptosis of H/R cardiomyocytes

To evaluate miR-195-5p’s protective effect on the heart in-depth, we established an H/R model in H9c2 cells to induce apoptosis of cardiomyocytes. The results revealed that compared with the BCG, the apoptosis rate of the H/R group and miR-NC group increased dramatically, the pro-apoptotic protein Bax was remarkably up-regulated, and the anti-apoptotic protein Bcl-2 was markedly down-regulated (*P*<0.05). Compared with the cells of the H/R group and miR-NC group, the rate of the H/R+miR-195-5p-mimics group decreased dramatically, the Bax was dramatically down-regulated, and the Bcl-2 was dramatically up-regulated (*P*<0.05) (Figure 3).

**Figure 3:** Effect of miR-195-5p overexpression on apoptosis of H/R myocardial cells (**A**) Effect of miR-195-5p overexpression on apoptosis rate of H/R cardiomyocytes. (**B**–**E**) Effect of miR-195-5p overexpression on apoptosis-related proteins (expression in H/R myocardial cells). *, # compared with BCG (*P*<0.05).

### miR-195-5p’s effect on TGF-β1/Smad3 signaling pathway in HF rats

Compared with the BCG and SOG, the TGF-β1 and Smad3 protein expression levels in HF rat myocardium increased dramatically (*P*<0.05), but those in the HF+miR-195-5p-agomir group decreased dramatically compared with the HF group (*P*<0.05). Online website of TargetScan7.2 predicted that there was a targeted relationship between miR-195-5p and Smad3. Hence, we conducted a dual-luciferase activity test and found that Smad3-3′UT Wt luciferase activity reduced obviously after miR-195-5p was overexpressed (*P*<0.05), but it had no effect on Smad3-3′UTR Mut luciferase activity (*P*>0.05). WB detection found that Smad3 protein expression in H9c2 cardiomyocytes reduced markedly after transfection of miR-195-5p-mimics (*P*<0.05) (Figure 4).

**Figure 4:** Effect of miR-195-5p on TGF-β1/Smad3 signaling pathway in HF rats (**A**) Effect of miR-195-5p on Smad3 dual luciferase reporter enzyme activity. (**B**) Effect of miR-195-5p on Smad3 protein expression in cardiomyocytes. (**C,D**) Effect of miR-195-5p on TGF-β1/Smad3 signaling pathway in HF rats. *, # compared with BCG (*P*<0.05).

### Effect of inhibiting TGF-β1/Smad3 signaling pathway on cardiomyocyte apoptosis

We inhibited the activation of TGF-β1/Smad3 signaling pathway by inhibiting Smad3 protein expression in H/R cardiomyocytes. Compared with the BCG, the Smad3 and TGF-β1 protein expression levels in the H/R group and Si-NC group were obviously up-regulated. When we down-regulated Smad3 protein expression in H/R cardiomyocytes, the Smad3 and TGF-β1 protein expression levels in the Si-Smad3 group cells were obviously down-regulated than that in the H/R group and Si-NC group (*P*<0.05). After detecting the cardiomyocyte apoptosis, we found that compared with the BCG, the apoptosis rate in the H/R group and Si-NC group increased dramatically, the pro-apoptotic protein Bax increased markedly, and the anti-apoptotic protein Bcl-2 decreased remarkably (*P*<0.05). Compared with the cells in the H/R group and Si-NC group, the rate in the Si-Smad3 group decreased markedly, the Bax decreased obviously, and the Bcl-2 increased dramatically (*P*<0.05) (Figure 5).

**Figure 5:** Effect of inhibiting TGF-β1/Smad3 signaling pathway on cardiomyocyte apoptosis (**A**) Inhibition of TGF-β1/Smad3 signaling pathway related protein expression in cardiomyocytes after Smad3. (**B**) Inhibitory effect of Smad3 on apoptosis rate of H/R cardiomyocytes. (**C**–**F**) Inhibitory effect of Smad3 on expression of apoptosis-related proteins in H/R cardiomyocytes. *, # compared with BCG (*P*<0.05).

## Discussion

HF is not only the final destination of most cardiovascular diseases, but also a complex clinical syndrome with new dysfunction caused by various diseases [2]. At present, HF is incurable clinically. Once confirmed, it will causes a heavy burden to the family and society [13]. It is the decompensation stage of cardiac insufficiency, and its main pathological basis is inflammatory reaction and cardiomyocyte apoptosis. Therefore, exploring the mechanism of HF inflammatory reaction and cardiomyocyte apoptosis is crucial for clinical prevention and treatment [2,14].

Recently, more and more miRNA are found to play a crucially regulatory part in HF [15]. As a vital miRNA, miR-195-5p has been verified to be effective in tumors in the past. For example, research [16] reported that it could inhibit cervical cancer cells’ migration and invasion by inhibiting ARL2. Recent studies [17] have found that it plays a crucially regulatory part in myocardial injury induced by high glucose, but its mechanism of action on cardiomyocytes has not been elaborated in detail. In our study, first, we established HF rat model by ligating abdominal aorta, and then we found that it expressed low in myocardium of HF rats. Previously, as to miRNA expression in heart during HF. Some studies [18] confirmed that miR-195-5p was down-regulated, which was consistent with our results. Its abnormal expression in HF rats made us guess that it might have certain influence on the occurrence and development of HF. Therefore, we up-regulated miR-195-5p expression in HF rats. The results revealed that when miR-195-5p was overexpressed, cardiac function of those rats had been dramatically improved, which was mainly reflected in the remarkable reduction of LVIDs, IVSd, IVSs, LVIDDD, and EF; those all responded to the systolic function and blood pumping function of the heart, and this was the main indicator of cardiac function [19]. Cardiomyocyte apoptosis is considered to be one of the main pathological mechanisms of HF, so we also used TUNEL method to test the apoptosis of cardiomyocytes in rats of each group. The results signified that its overexpression could reduce the apoptosis rate of cardiomyocytes in those rats significantly. Bax and Bcl-2 belong to the Bcl family. The proportion of bcl2/bax determines the apoptosis of cells [20]. However, the increase of Cle-Caspase-3 activity is generally considered as a sign of apoptosis and a positive indicator of cancer treatment efficacy [21]. At the same time, we also observed that miR-195-5p could reduce the Bax and activated Cle-Caspase-3 expression levels and up-regulate Bcl-2 expression, which further manifested that it could reduce the apoptosis of cardiomyocytes in HF rats.

To verify miR-195-5p’s effect on cardiomyocyte apoptosis in depth, we established an H/R cell model to induce cardiomyocyte apoptosis and up-regulated miR-195-5p expression. As a result, we also observed that its expression could obviously inhibit hypoxia-induced cardiomyocyte apoptosis, which was consistent with our results in *in vivo* experiments. Although its effect on cardiomyocyte apoptosis has not been studied in detail in the past, many studies have been conducted on the effect of miRNA on cardiomyocyte apoptosis. For example, some studies [22] have reported that miR-9 can inhibit hypoxia-induced cardiomyocyte apoptosis by targeting Yap1. Another study [23] has pointed out that miR-486 can regulate apoptosis of cardiomyocytes by regulating Bcl-2. All these studies have proved the role of miRNA in cardiomyocyte apoptosis, and also explored and elaborated its mechanism. Nevertheless, miR-195-5p’s mechanism on cardiomyocyte apoptosis is still unclear. TGF-β1/Smad3 signaling pathway has been proved to be tied to the occurrence and development of various diseases in the past, including HF. Previous studies [24] have reported that angiotensin II can stimulate the apoptosis of cardiomyocytes in HF rats by regulating this pathway. We found a targeted relationship between miR-195-5p and Smad3 through online website prediction, and Smad3 is one of the key factors in this pathway. Previous studies [25] have reported that miR-132 can induce cardiomyocyte apoptosis in HF by regulating Smad3. In our research, we also found that this signaling pathway was dramatically activated in HF rats. But when we up-regulated miR-195-5p expression, we found that this pathway was markedly inhibited, which suggested that miR-195-5p could inhibit the activation of this pathway, and we also verified the targeted relationship between miR-195-5p and Smad3 with dual-fluorescein reporter enzyme. Ultimately, in order to prove that miR-195-5p may indeed exert its effect on HF by regulating this pathway, we also down-regulate the Smad3 protein expression in cardiomyocytes to inhibit this pathway. The results showed that when we inhibited this pathway, the apoptosis rate of cardiomyocytes induced by H/R reduced obviously, and the Bax and activated Cle-Caspase-3 protein expression levels reduced dramatically, but the Bcl-2 protein expression increased greatly. Research [26] has also confirmed that the apoptosis rate of cardiomyocytes can be reduced by inhibiting this pathway in HF mouse model. This also confirms our conclusion.

Overall, miR-195-5p can inhibit cardiomyocyte apoptosis in HF rats by regulating TGF-β1/Smad3 signaling pathway, improve cardiac function in HF rats, and may become a potential target for HF therapy. However, there are still some limitations in the present study. On the one hand, it is not clear whether miR-195-5p has other targets on those rats. On the other hand, the possible downstream mechanism of TGF-β1/Smad3 is not clear. We will conduct further in-depth research in future experiments to elaborate miR-195-5p’s mechanism on HF at length.

## Conclusion

Overall, miR-195-5p can inhibit cardiomyocyte apoptosis in HF rats by regulating TGF-β1/Smad3 signaling pathway, improve cardiac function in HF rats, and may become a potential target for HF therapy. However, there are still some limitations in the present study. On the one hand, it is not clear whether miR-195-5p has other targets on those rats. On the other hand, the possible downstream mechanism of TGF-β1/Smad3 is not clear. We will conduct further in-depth research in future experiments to elaborate miR-195-5p’s mechanism on HF at length.

## Abbreviations

ARL2: ADP ribosylation factor like GTPase 2
Bax: BCL2 associated X, apoptosis regulator
BCG: blank control group
Bcl-2: BCL2 apoptosis regulator
EF: ejection fraction
FBS: fetal bovine serum
HF: heart failure
H/R: hypoxia/reoxygenation
IVSd: interventricular septal end-diastolic
IVSs: interventricular septal end-systolic
LVIDd: left ventricular end-diastolic inner diameter
LVIDs: left ventricular end-systolic inner diameter
LVIDDD: left ventricular end-diastolic diameter
LSD: lysergic acid diethylamide
NC: negative control
PI: propidium iodide
SD rats: sprague dawley rats
Smad: signal transduction protein
TGF-β1: transforming growth factor-β1
TUNEL: terminal deoxynucleotidyl transferase dUTP nick end labeling
WB: western blotting
